The article "Resting-State Functional Magnetic Resonance Image to Analyze Electrical Biological Characteristics of Major Depressive Disorder Patients with Suicide Ideation" was published in 2022. Journal: Comput Math Methods Med.

# Resting-State Functional Magnetic Resonance Image to Analyze Electrical Biological Characteristics of Major Depressive Disorder Patients with Suicide Ideation

**DOI:** 10.1155/2022/3741677

**Published:** 2022-06-13

**Authors:** Cui He, Yeyan Wang, Hanping Bai, Ruiting Li, Xiangming Fang

**Affiliations:** ^1^Department of Psychiatry, Wuhan Youfu Hospital, Wuhan, 430023 Hubei, China; ^2^Mental Depression Centre, Renmin Hospital of Wuhan University, Wuhan, 430205 Hubei, China

## Abstract

The study was aimed to explore the brain imaging characteristics of major depressive disorder (MDD) patients with suicide ideation (SI) through resting-state functional magnetic resonance imaging (rs-fMRI) and to investigate the potential neurobiological role in the occurrence of SI. 50 MDD patients were selected as the experimental group and 50 healthy people as the control group. The brain images of the patients were obtained by MRI. Extraction of EEG biological features was from rs-fMRI images. Since MRI images were disturbed by noise, the initial clustering center of FCM was determined by particle swarm optimization algorithm so that the noise of the collected images was cleared by adaptive median filtering. Then, the image images were processed by the optimized model. The correlation between brain mALFF and clinical characteristics was analyzed. It was found that the segmentation model based on the FCM algorithm could effectively eliminate the noise points in the image; that the zALFF values of the right superior temporal gyrus (R-STG), left middle occipital gyrus (L-MOG), and left middle temporal gyrus (L-MTG) in the observation group were significantly higher than those in the control group (*P* < 0.05); and that the average zALFF values of left thalamus (L-THA) and left middle frontal gyrus (L-MFG) decreased. The mean zALFF values of L-MFG and L-SFG demonstrated good identification value for SI in MDD patients. In summary, MRI images based on FCM had a good convergence rate, and electrical biological characteristics of brain regions were abnormal in MDD patients with SI, which can be applied to the diagnosis and treatment of patients with depression in clinical practice.

## 1. Introduction

Major depressive disorder (MDD) is a chronic mental disorder of a high incidence. MDD patients have a high rate of suicide. Its clinical manifestations include lack of interest, persistent depressive mood, and anhedonia [1]. Suicide ideation (SI) refers to the behavior that patients have thoughts of ending their own lives. Relevant studies show that 40%-70% of depressed patients have SI [2–5]. From the perspective of social psychology, many studies have explored the early signs of SI of MDD patients and predicted the risk factors of suicide, but it is highly subjective and there are few reproducible biological indicators [6, 7]. In recent years, brain imaging studies have found that MDD patients with SI have obvious brain function impairment and many studies have shown that the biological phenotype of SI in MDD patients is related to brain structure and function [8, 9].Magnetic resonance imaging (MRI) is widely used in diagnosis of stroke patients and monitoring of brain function in clinical rehabilitation therapy because it does not cause ionizing radiation to human body and can clearly present soft tissue conditions [10]. Functional MRI (fMRI) has applications in the detection of brain network neural function, which is mainly divided into resting-state (RS-FMRI) and task-state fMRI. fMRI research methods include near-infrared spectroscopy, cerebral magnetic resonance spectrum analysis, and other magnetic resonance technologies [11]. The resting state refers to the state in which the subject is awake without deliberate thought acquisition, and in relaxation and stillness. Studies have shown that there are still spontaneous local neural activities in the brain at this time [11]. MDD patients with SI have abnormal changes in bilateral middle occipital gyrus function [12, 13], and the specific mechanism of abnormal changes in brain imaging is not clear.

Fuzzy C-means clustering (FCM) algorithm has broad applications in pattern recognition, image processing, and fuzzy modeling. It can optimize the segmentation method of brain MR image. Despite the simple design, FCM can achieve better classification effect in dealing with multiple classification problems [14]. Nowadays, FCM has been widely used in medical diagnosis, image analysis, agricultural environmental engineering, target recognition, and other aspects. Especially, image processing can reduce image noise, which has important guiding significance for the analysis and research of imaging images.

Current studies show that MDD patients with SI have obvious brain function impairment, mainly the three core brain network injuries. Local consistency indicators of rs-fMRI brain images have good stability and high repeatability, and patients have good compliance with it, effectively avoiding potential confounding factors in MRI [15]. MRI studies showed that the synergy of multiple brain areas can trigger MDD in patients with SI, but there are few related studies on it. In this study, the FCM algorithm was used to optimize the segmentation method of brain MRI image, to compare brain structure and function difference in MDD patients with and without SI and track characteristics of brain function change, and expected to provide a theoretical basis for the prevention of SI in MDD patients.

## 2. Materials and Methods

### 2.1. Clinical Data

In the study, 50 patients with MDD admitted to the hospital from March 2020 to June 2021 were selected. All patients met the MDD diagnostic criteria of *the Third Edition of Chinese Classification and Diagnostic Criteria for Mental Disorders* [16], and their 24-item scores of Hamilton Depression (HAMD) were all ≥20 points. All 50 patients were at the first onset, aged 18-56 years and averaged 37.2 ± 11.3 years. The course of disease was 0.09-3 years, with an average of 1.6 ± 1.9 years. (HAMD24) scores ranged from 35 to 68, with an average of 42.1 ± 7.3. A total score of 20 or more was considered mild or moderate depression, and a score of 35 or more was considered major depression. After systematic training, the scale was evaluated and recorded by a specialized physician in the psychiatric department. The patients' compliance when filling out the scale was analyzed for the reliability of later scale scores. 50 healthy people who underwent physical examination in the same period were selected as the control group according to the principle that race, age, sex, and educational level were close to those of the observation group. The Beck Suicide Ideation Scale was selected for the evaluation of SI. All the patients who fully met the inclusion criteria accepted the test regulations and signed the informed consent form. This study was approved by the ethics committee of hospital.

The inclusion criteria is as follows: (I) first onset; (II) basic vital signs were stable, capable of language expression and conscious; (III) no history of head injury; (IV) no nervous system diseases and other mental disorders; (V) no physical disease, alcohol, visual impairment, and MRI contraindications; and (VI) those who were used to use the right hand in test. The exclusion criteria are as follows: (I) with a history of drug dependence, abuse, and alcoholism; (II) past manic episodes; (III) psychogenic depression; (IV) unable to accept MRI examination due to his own reasons; and (V) the clinical data was imperfect.

### 2.2. MRI Scanning Equipment and Parameter Setting

3.0 T magnetic resonance imaging system was used, and the coils used are standard 12-channel head coils. When scanned, the subjects were awake, lied flat on the examination bed, and kept their limbs relaxed and their heads stable, closed their eyes, and breathed evenly. They wore the anti-noise headphones to reduce the influence of noise on the experiment so that the experiment can be officially started when the subjects were in a calm state. Radiology professionals should evaluate the safety of instruments before data acquisition. Then, the inspection process and precautions were explained in detail to the patients. Scanning sequence includes conventional MRI head plain scanning sequence and static BOLD-fMRI scanning single excitation echo planar imaging, with parameters as follows.

In Rs-fMRI imaging, the scanning mode is axial scanning, using a single excitation gradient echo-plane echo sequence, with the following scanning parameters: fa = 90, TE = 40 MS, FOV = 24 cm × 24 cm, TR = 2000 MS, matrix 64 × 64, thickness/spacing = 4.0/0 mm, and scanning time = 8.

During the scan, the patient was required to keep the heads still as much as possible, and the image data that did not meet the requirements, such as the image data with large head movement range, was removed. Every step of data processing should ensure data quality and avoid mixed adverse factors such as noise.

### 2.3. FCM Algorithm

Clustering analysis is a mathematical method to classify similar data in a sample set according to a specific criterion, that is, according to similarity criteria, a group of vectors of category markers in a specific space are divided into several subsets. The steps of clustering include the following: (I) feature extraction and selection of clustered objects; (II) to define similarity measure function; (III) clustering; and (IV) evaluation of results. FCM depends on the selection of initial clustering center to a great extent. When the initial clustering center deviates from the global optimal clustering center seriously, the algorithm will fall into local minimum. The flow chart of the FCM algorithm is shown in Figure 1. First, initialize the cluster center and membership matrix. Then, calculate cluster centers, update membership matrix, and output cluster center.

### 2.4. Evaluation Criteria of Images Segmented by the FCM Algorithm

I algorithm setting and parameter optimization, index *m* (*m* = 2) of membership matrix *u*, maximum iteration times *T*(*T* = 100), and iteration termination condition *ε* (*ε* = 0.0001); II the initial clustering center of FCM is obtained by PSO algorithm; III filtering all acquired images; IV according to the formula, the cluster center IS continuously updated; V the iteration process is stopped if satisfactory results can be obtained by clustering or if the number of iterations k > T. Otherwise, return to the previous step; and VI according to the finally obtained membership matrix, the pixel size required by the target is set to the value of a corresponding cluster center, and the obtained MRI image can be segmented.

The effect of MRI image segmentation was evaluated using the Jaccard similarity coefficient (JaccardSimilarity, JS). The JS equation was shown as follows:

(1) $$\begin{array}{c} JS=\frac{\left|S_{1}\cap S_{2}\right|}{\left|S_{1}\cup S_{2}\right|}, \end{array}$$

where *S*_1_ represents the region to be segmented, *S*_2_ represents the ground truth, and a higher JS value indicates better clustering performance of the algorithm, which also means higher the segmentation accuracy of the algorithm.

### 2.5. FMRI Data Preprocessing

The fMRI data is processed by data processing assistant for RS-fmri advanced edition (DPARSFA) software on Matlab platform. The specific process is as follows: (I) format conversion is required to transform from digital imaging and communications medicine (DICOM) to neuroimaging informatics technology initiative (NIFTI); (II) head movement correction; (III) spatial standardization: brain fMRI images are standardized in terms of image size and direction; and (IV) time correction. As for the interval scanning of rsfMRI, time correction is required to correct scanning time difference to eliminate the inconsistency of scanning time of adjacent layers: (V) space smoothing and (VI) filtering. The first 15 time points are eliminated to remove the influence of unstable initial time series; and (VII) regression covariates. It refers to covariates such parameters as brain mean signal, head movement parameters, cerebrospinal fluid signal, and white matter signal. Images that rotate more than 3° and translate more than 3 mm are eliminated. According to the template of nerve research in Montreal, Canada, the brain shape differences are eliminated. The 3D-T1 anatomical image with high resolution is segmented into consistent gray matter, white matter, and cerebrospinal fluid. The functional anatomical information of the image is based on the information obtained from structural image segmentation and registered to MNI spatial template. The standardized image needs to be resampled and then mapped to the standard brain.

The ALFF analysis uses the REST1.9 software of Matlab platform for data analysis. For image data after linear drift removal and low frequency filtering (0.01-0.08 Hz), the whole brain signal is converted to a frequency domain power spectrum by fast Fourier transform. The area under the peak of the power spectrum can be regarded as the energy of the signal. After calculation, the average value of each voxel in the frequency signal amplitude is obtained. The ALFF value is normalized by *Z*-score transformation, and the signal difference is eliminated. The zALFF statistical analysis of each voxel obtained after *z* transformation is as follows:

(2) $$\begin{array}{c} \text{Zscore}=\frac{\text{ALFF}-\text{mALFF}}{\text{SD}}. \end{array}$$

*SD* represents the standard deviation of ALFF values of all voxels in the whole brain. *mALFF* represents the ALFF value of each voxel divided by the whole brain signal amplitude.

### 2.6. Statistical Methods

SPSS22.0 was used to process the experimental data, and analysis methods were selected according to different situations. Univariate analysis and Chi-square test (*χ*2 test) were used to compare the counting data between groups, and the mean ± standard scale was used for the measurement data. *P* < 0.05 meant that there were statistical differences.

## 3. Results

### 3.1. Clinical Data of Subjects

Table 1 showed the clinical data of the two groups in this study. In the SI group, there were 50 cases, including 26 males and 24 females, with an average age of 37.2 ± 11.03 points; in the control group, there were 20 males and 30 females. The statistical results showed that there was no significant difference in gender, age, and years of education between the two groups. The HAMD score and SI degree were significantly different between the two groups.

### 3.2. Comparison of Fitness Function Values of Algorithms

The fitness function value of the FCM algorithm was compared with that of the traditional PSO FCM algorithm, as shown in Figure 2. The average value and the worst solution of FCM were both higher than those of the traditional PSO FCM.  Figure 3 showed the convergence speed of the FCM image segmentation algorithm, and the results show that the algorithm proposed in this study converged to the optimal solution quickly.

### 3.3. rs-fMRI Images

In Figure 4, the image was from a 46-year-old male patient. In Figure 4(a), 181 × 140 pixels were selected manually and segmented by the FCM algorithm, and the results are shown in Figure 4(b). It was noted visually that the selected KFCM segmentation method proposed in this study can eliminate the noise points in the image and had good noise robustness. Figure 4(a) showed many noises with no obvious morphology. Figure 4(b) showed that the noise was reduced and the shape was obvious.

### 3.4. Brain MRI Images

In Figure 5, the image was from a 52-year-old female patient. Brain MRI images of patients were processed by the FCM algorithm, and white matter and gray matter are segmented in Figure 5.

### 3.5. mALFF Value of the Brain Region

Seven Regions of Interests (ROIs) were selected, namely, the right superior temporal gyrus (R-STG), left angular gyrus (L-AG), left thalamus (L-THA), left middle occipital gyrus (L-MOG), left middle frontal gyrus (L-MFG), left superior frontal gyrus (L-SFG), and left middle temporal gyrus (L-MTG). As shown in Figure 6, the zALFF value of R-STG, L-MOG, and L-MTG in the observation group was significantly higher than that in the control group (*P* < 0.05) and that the zALFF average value of L-THA and L-MFG decreased.

### 3.6. ROC Curve Analysis

ROC curve was used to analyze the average zALFF value of the brain RoI and evaluate the SI degree in patients. As shown in Figure 7, zALFF = 0.677 of R-STG had a sensitivity of 82.4% and specificity of 46.2%. The area under the curve of L-AG was 0.826, and the sensitivity and specificity were 85.6% and 55.8%, respectively, when the cut-off point was zALFF = 0.788. The sensitivity and specificity of zALFF = 0.778 for L-MOG were 85.9% and 46.2%, respectively. The sensitivity and specificity of L-MFG were 72.6% and 83.5%, respectively. The sensitivity and specificity of zALFF = 0.762 for L-MTG were 65.8% and 65.9%, respectively. As shown in Figures 8 and 9, the zALFF average values of L-MFG and L-SFG had good identification value for SI in MDD patients.

### 3.7. Brain Region Location

Figure 10 showed the locations of L-SFG, L-MFG, L-AG, and R-STG in the brain area, expressed by purple marks in the red box.

## 4. Discussion

MDD is a common mental disorder related to suicide. Relevant data show that the lifetime suicide rate of MDD patients is 2%-12%, which has become a serious social problem and brings great damage to the economy. At present, the brain neurobiological mechanism of MDD patients is not completely clear, and there is a lack of specificity of SI. The diagnosis of MDD indicates SI. Suicide is driven by MDD symptoms and neurobiological processes [17]. Functional neuroimaging has shown that patients with MDD have reduced hemodynamic excitation in the prefrontal region [18, 19]. Lan et al. (2019) [20] showed that, compared with MDD patients without SI, low-frequency oscillating amplitude ALFF values in the right hippocampus, bilateral thalamus, and caudate nucleus of juvenile MDD patients with SI increased. The research results of Pan et al. (2020) [21] showed that repetitive transcranial magnetic stimulation may be a method to treat severe depressive disorder, which can quickly reduce SI and environmental MDD. In this study, the brain imaging features of SI were investigated, and the images were processed using an ion group optimization algorithm. Compared with controls, MDD patients had mean zALFF in the left thalamus (L-THA) and left middle frontal gyrus (L-MFG). The value was significantly higher than that of the control group (*P* < 0.05), which was consistent with the findings of Lan et al. Mean zALFF values of L-MFG and L-SFG showed good SI identification value in MDD patients.

fMRI is a new imaging diagnostic method, which is noninvasive, dynamic, and objective and has great advantages in evaluating brain functional activities and functional connections. fMRI can also study brain functional activities in vivo, combined with brain emotional activities. Further analysis of the relationship between brain dysfunction and cognition in MDD patients with SI is of great significance for early detection, prevention, and intervention of suicidal behavior in MDD patients [22]. fMRI imaging studies have shown that there is a difference in activation models in the cerebellar, goblin, and buckle back and the decreased functional connections of R-STG, L-AG, L-THA, L-MOG, L-MFG, L-SFG, and L-MTG and increased motion function connections are associated with suicide behavior [23]. Extensive network abnormalities have been noted in rs-FMRI studies of MDD patients. Cao and Chen (2016) [12] used rs-fMRI technology to study MDD patients and found that low-frequency amplitude of *Z* in L-STG and R-MFG of MDD patients with SI significantly decreased and that neural abnormalities in the frontal lobe may be associated with suicidal tendencies in adolescents with MDD. rs-fMRI is an important way to study the spontaneous brain functional activities of the human brain in the resting state. It uses non-external stimulation to analyze the internal signal oscillations due to the irritation. Spontaneous activity of brain neurons in resting state leads to low-frequency oscillation of local BLOD signal [23]. Zhang et al. (2020) [24] found that the reduction of left DLPFC in MDD patients was associated with SI. This study found that MDD was more likely to occur in lesions located in the anterior circulation region, left hemisphere, frontal lobe, and temporal lobe and that zALFF average values of L-MFG and L-SFG demonstrated good identification value for SI in MDD patients. The damage of frontal and temporal lobes may be the biological basis of SI in MDD patients. FCM is a clustering algorithm capable of organizing various datasets and obtaining accurate classifications. Zhang et al. (2020) [25] using FCM and PSO hybrid clustering can significantly improve the convergence speed and clustering effect. In this study, the brain MRI images of MDD patients were processed by the FCM algorithm, and the intelligent algorithm could segment white matter and gray matter, the organs can remove noise points in the image, and the MRI image based on FCM has a good convergence speed.

## 5. Conclusion

In this study, an FCM algorithm was introduced to segment rs-fMRI images of MDD patients and analyzed the correlation of mALFF and clinical characteristics in the brains of MDD patients and healthy controls. The results show that the image segmentation algorithm based on FCM can quickly converge to the optimal solution and the computational complexity is greatly reduced compared with the traditional FCM algorithm. The mean zALFF values of the left thalamus (L-THA) and left middle frontal gyrus (L-MFG) were significantly higher than those of the control group (*P* < 0.05). The mean zALFF values of L-MFG and L-SFG showed good identification value in MDD patients with cognitive impairment in brain white matter nerve fibers.

However, some limitations should be noted in the study. Image segmentation involves a wide range of content, images in various fields are very different, and the scope of use is also limited. The small sample size reduces the power of the study. In the follow-up, it is necessary to expand the sample size to strengthen the research results and to continuously improve the nerve fiber detection technology, to further explore the function of various brain regions, and to better understand the role of pathway impairment on cognition.

## Figures and Tables

**Figure 1:** Flowchart of the FCM algorithm.

**Figure 2:** Fitness function value.

**Figure 3:** Convergence speed of FCM algorithm.

**Figure 4:** rs-fMRI images.

**Figure 5:** Segmentation results.

**Figure 6:** Statistical analysis of interested brain time series between the two groups. ∗Compared with the control group, *P* < 0.05.

**Figure 7:** The area under ROC curve and the demarcation point distribution.

**Figure 8:** The specificity and sensitivity of the ROC curve for MDD patients with SI.

**Figure 9:** ROC analysis results of brain areas.

**Figure 10:** ROI locations of brain regions.

**Table 1:** Statistics of clinical data.

Item	Control group	SI group	*P*
Gender (male/female)	26/24	20/30	0.068^a^
Age (years)	42.2 ± 9.12	37.2 ± 11.03	0.142^b^
SI degree (score)	—	1.84 ± 0.08	—
HAMD score	—	39.38 ± 2.18	—
Years of education (score)	9.82 ± 0.29	9.86 ± 0.32	0.083
Number of previous suicides	—	2.93 ± 2.03	—

Note: ^a^Chi-square test; ^b^analysis of variance.

## Data Availability

The data used to support the findings of this study are available from the corresponding author upon request.

## References

[1] Ducharme S., Dols A., Laforce R. (2020). Recommendations to distinguish behavioural variant frontotemporal dementia from psychiatric disorders. *Brain*.

[2] Wagner G., Li M., Sacchet M. D. (2021). Functional network alterations differently associated with suicidal ideas and acts in depressed patients: an indirect support to the transition model. *Translational Psychiatry*.

[3] Kim K., Shin J. H., Myung W. (2019). Deformities of the globus pallidus are associated with severity of suicidal ideation and impulsivity in patients with major depressive disorder. *Scientific Reports*.

[4] Li J., Duan X., Cui Q., Chen H., Liao W. (2019). More than just statics: temporal dynamics of intrinsic brain activity predicts the suicidal ideation in depressed patients. *Psychological Medicine*.

[5] Basta M., Micheli K., Karakonstantis S. (2021). Suicidal ideation in adolescents and young adults in Greece: prevalence and association with sociodemographic variables, mental health and substance use. *European Child & Adolescent Psychiatry*.

[6] Sun Y., Blumberger D. M., Mulsant B. H. (2018). Magnetic seizure therapy reduces suicidal ideation and produces neuroplasticity in treatment-resistant depression. *Translational Psychiatry*.

[7] Dolsen M. R., Cheng P., Arnedt J. T. (2017). Neurophysiological correlates of suicidal ideation in major depressive disorder: Hyperarousal during sleep. *Journal of Affective Disorders*.

[8] Greer N., Ackland P., Sayer N. (2019). *Relationship of deployment-related mild traumatic brain injury to posttraumatic stress disorder, depressive disorders, substance use disorders, suicidal ideation, and anxiety disorders: a systematic review [Internet]*.

[9] Proctor C. J., Best L. A. (2019). Social and psychological influences on satisfaction with life after brain injury. *Disability and Health Journal*.

[10] Yu X., Yang L., Song R. (2017). Changes in structure and perfusion of grey matter tissues during recovery from ischaemic subcortical stroke: a longitudinal MRI study. *The European Journal of Neuroscience*.

[11] Dichter G. S., Gibbs D., Smoski M. J. (2015). A systematic review of relations between resting-state functional-MRI and treatment response in major depressive disorder. *Journal of Affective Disorders*.

[12] Cao J., Chen X., Chen J. (2016). Resting-state functional MRI of abnormal baseline brain activity in young depressed patients with and without suicidal behavior. *Journal of Affective Disorders*.

[13] Chen V. C., Kao C. J., Tsai Y. H., Cheok M. T., McIntyre R. S., Weng J. C. (2021). Assessment of disrupted brain structural connectome in depressive patients with suicidal ideation using generalized Q-sampling MRI. *Frontiers in Human Neuroscience*.

[14] Hu M., Zhong Y., Xie S., Lv H., Lv Z. (2021). Fuzzy system based medical image processing for brain disease prediction. *Frontiers in Neuroscience*.

[15] Li H., Chen Z., Gong Q., Jia Z. (2020). Voxel-wise meta-analysis of task-related brain activation abnormalities in major depressive disorder with suicide behavior. *Brain Imaging and Behavior*.

[16] Zhou T., Thung K. H., Liu M., Shi F., Zhang C., Shen D. (2020). Multi-modal latent space inducing ensemble SVM classifier for early dementia diagnosis with neuroimaging data. *Medical Image Analysis*.

[17] Rotenstein L. S., Ramos M. A., Torre M. (2016). Prevalence of depression, depressive symptoms, and suicidal ideation among medical students: a systematic review and meta-analysis. *JAMA*.

[18] Croarkin P. E., Nakonezny P. A., Deng Z. D. (2018). High-frequency repetitive TMS for suicidal ideation in adolescents with depression. *Journal of Affective Disorders*.

[19] Hedley D., Uljarević M., Foley K. R., Richdale A., Trollor J. (2018). Risk and protective factors underlying depression and suicidal ideation in autism Spectrum disorder. *Depression and Anxiety*.

[20] Lan M. J., Rizk M. M., Pantazatos S. P. (2019). Resting-state amplitude of low-frequency fluctuation is associated with suicidal ideation. *Depress Anxiety*.

[21] Pan F., Shen Z., Jiao J. (2020). Neuronavigation-guided rTMS for the treatment of depressive patients with suicidal ideation: a double-blind, randomized, Sham‐controlled trial. *Clinical Pharmacology & Therapeutics*.

[22] Rizk M. M., Rubin-Falcone H., Lin X. (2019). Gray matter volumetric study of major depression and suicidal behavior. *Psychiatry Research: Neuroimaging*.

[23] Chen M. H., Lin W. C., Tu P. C. (2019). Antidepressant and antisuicidal effects of ketamine on the functional connectivity of prefrontal cortex-related circuits in treatment-resistant depression: a double-blind, placebo-controlled, randomized, longitudinal resting fMRI study. *Journal of Affective Disorders*.

[24] Zhang R., Wei S., Chang M., Jiang X., Tang Y., Wang F. (2020). Dorsolateral and ventrolateral prefrontal cortex structural changes relative to suicidal ideation in patients with depression. *Acta Neuropsychiatrica*.

[25] Zhang J., Ma Z. (2020). Hybrid fuzzy clustering method based on FCM and enhanced logarithmical PSO (ELPSO). *Computational Intelligence and Neuroscience*.

